The article "Therapeutic Effects of the Proximal Femoral Nail for the Treatment of Unstable Intertrochanteric Fractures" was published in 2022. Journal: Evid Based Complement Alternat Med.

# Therapeutic Effects of the Proximal Femoral Nail for the Treatment of Unstable Intertrochanteric Fractures

**DOI:** 10.1155/2022/1001354

**Published:** 2022-09-02

**Authors:** Yuwei Cai, Wenjun Zhu, Nan Wang, Zhongxiang Yu, Yu Chen, Shengming Xu, Juntao Feng

**Affiliations:** ^1^Department of Orthopedics, Shuguang Hospital Affiliated to Shanghai University of Traditional Chinese Medicine, Shanghai 200120, China; ^2^Department of Traditional Chinese Medicine, Shanghai YangZhi Rehabilitation Hospital (Shanghai Sunshine Rehabilitation Center), School of Medicine, Tongji University, Shanghai 201619, China

## Abstract

**Objective:**

The aim of this study was to analyze the clinical effect of the proximal femoral nail on elderly patients with unstable intertrochanteric fracture and the effect of the proximal femoral nail on serum levels of matrix metalloproteinases (MMPs) and osteoprotegerin (OPG).

**Methods:**

The elderly patients with unstable intertrochanteric fracture of the femur admitted to our hospital from January 2017 to January 2021 were studied. 100 patients were randomly divided into two groups: the control group (*n* = 50) and the observation group (*n* = 50). The patients in the control group were treated with a proximal femoral locking compression plate. The patients in the observation group were treated with the proximal femoral antirotation intramedullary nail. The clinical therapeutic effects of the two groups and the changes in serum MMPs and OPG levels before and after treatment were analyzed.

**Results:**

Compared with the control group, the operation time, postoperative landing time, and fracture healing time of the observation group were significantly shortened, and intraoperative blood loss was significantly reduced (*P* < 0.05). Compared with the control group, the total effective rate of patients in the observation group was significantly higher (*P* < 0.05). After treatment, the levels of CRP, IL1*β*, IL2, MMP-2, MMP-6, TIMP-1, and RANKL decreased significantly in both groups (*P* < 0.05), while the levels of OPG increased significantly (*P* < 0.05). Compared with the control group, the changes in the above indexes were more obvious in the observation group (*P* < 0.05).

**Conclusion:**

The proximal femoral antirotation intramedullary nail has a better therapeutic effect on elderly patients with unstable intertrochanteric fracture, and the level of MMPs and OPG may be related to the treatment process.

## 1. Introduction

Intertrochanteric fractures of the femur are common surgical fractures with high morbidity rates [1, 2]. In order to improve the mobility of the lower extremities and improve the prognosis of patients, patients with intertrochanteric fractures should receive immediate surgery and actively perform lower extremity functional exercises [3]. The proximal femoral anti-rotation intramedullary nail is a common method for the treatment of femoral intertrochanteric fractures, with the advantages of less trauma and easy operation [4]. Matrix metalloproteinases (MMPs) regulate the remodeling process of the extracellular matrix and are also widely involved in the process of bone tissue injury and healing [5]. The receptor activator of nuclear factor kappa B ligand/osteoprotegerin (RANKL/OPG) is a key signal transduction pathway of bone metabolism and is closely related to the pathological and physiological processes of bone tissue [6]. However, there is no relevant report on the level of MMPs during the treatment of elderly unstable intertrochanteric fractures with proximal femoral antirotation intramedullary nails. This study analyzed the clinical effect of the proximal femoral antirotation intramedullary nail on elderly patients with unstable intertrochanteric fractures and the effect on serum levels of MMPs and OPG in order to provide a reference for clinical treatment.

The article "Therapeutic Effects of the Proximal Femoral Nail for the Treatment of Unstable Intertrochanteric Fractures" was published in 2022. Journal: Evid Based Complement Alternat Med.

## 2. Materials and Methods

### 2.1. Research Objects

Elderly patients with unstable femoral intertrochanteric fractures admitted to our hospital from January 2017 to January 2021 were selected as the research subjects. Inclusion criteria were as follows: all patients met the diagnostic criteria for unstable intertrochanteric fractures [7] and were diagnosed by X-ray; there is a clear history of trauma; hip pain, swelling, lower extremity dysfunction; patient has severe lower extremity deformity and valgus, and local tenderness is obvious; clinical data are complete. Exclusion criteria are as follows: combined with severe bone disease; severe metabolic dysfunction; patients with concurrent malignant tumors; patients taking drugs that affect bone metabolism within the past 3 months; patients with incomplete clinical data or who disagree with this study. 100 patients were randomly divided into two groups according to the treatment method. Control group (*n* = 50): 24 males and 26 females; aged 61–72 years, mean 66.5 ± 8.5 years old; 28 patients with EvansIII (intertrochanteric fractures combined with greater trochanteric fractures with displacement, no posterolateral support, and comminuted posterior fracture); and 22 patients with EvansIV (combined lesser trochanter fracture with displacement and no medial support). Observation group (*n* = 50): 23 males and 27 females; aged 61–72 years, mean 66.8 ± 8.8 years old; 29 patients with EvansIII; and 21 patients with EvansIV. There was no statistical difference in general data such as gender and average age between the two groups (*P* > 0.05).

The article "Therapeutic Effects of the Proximal Femoral Nail for the Treatment of Unstable Intertrochanteric Fractures" was published in 2022. Journal: Evid Based Complement Alternat Med.

### 2.2. Treatment Methods

The patients in the control group were treated with the proximal femoral locking compression plate. The patients were in a supine position, continuous epidural anesthesia was administered, a soft pillow was placed on the affected buttocks, and the surgical incision was selected at 2.9 ± 1 cm above the apex of the greater trochanter, extending laterally. Separate the skin and subcutaneous tissue of the patient, expose the fracture end, use Kirschner wire fixation after satisfactory reduction and traction, insert screw-type screws through C-arm fluoroscopy, lock the screws at the distal end, and move the affected limb.

The patients in the observation group were treated with the proximal femoral antirotation intramedullary nail. The patients were in a supine position, continuous epidural anesthesia was administered, adduction of the affected limb about 15° in neutral position, reduction under C-arm fluoroscopy, and longitudinal incision about 1 cm above the greater trochanter, and an open 5.5 ± 0.5 cm. The needle was placed at the apex of the tuberosity, and after reaming, the proximal antirotation intramedullary nail was inserted and screwed into the helical blade and distal locking nail.

### 2.3. Observation Indicators and Methods

#### 2.3.1. Analysis of Clinical Treatment Effect of the Two Groups of Patients

In this study, the operation time, intraoperative blood loss, postoperative landing time, and fracture healing time of the two groups of patients were analyzed, and the total effective rate of the treatment was also analyzed. The treatment effect is divided into four categories. Cure: at the follow-up after 12 months of treatment, the Harris score of the hip joint of the patient is more than 90 points. Significant effect: at the follow-up after 12 months of treatment, the Harris score of the hip joint of the patient is more than 80 points. Valid: at the follow-up after 12 months of treatment, the Harris score of the hip joint of the patient is more than 70 points. Invalid: at the follow-up after 12 months of treatment, the Harris score of the hip joint of the patient is not more than 70 points. Total effective rate = (cure + significantly effect + valid)/total number of cases × 100%.

#### 2.3.2. Biochemical Index Analysis

Before and after treatment, 5 ml of fasting venous blood was collected in the morning. Serum MMPs (including MMP2, MMP6, and its inhibitor TIMP1), RANKL/OPG levels, CRP, Interleukin (IL)1*β,* and IL2 before and after treatment were analyzed by enzyme-linked immunosorbent assay. MMP2 and MMP6 detection kits were purchased from Cell Signaling. TIMP1 detection kit was purchased from R&D company. RANKL detection kit was purchased from Santa Cruz company. The OPG, CRP, IL1*β,* and IL2 detection kit was purchased from Abcam Company. All detection operations were performed in accordance with the kit instructions.

The article "Therapeutic Effects of the Proximal Femoral Nail for the Treatment of Unstable Intertrochanteric Fractures" was published in 2022. Journal: Evid Based Complement Alternat Med.

#### 2.3.3. Patient Follow-Up

All patients were followed up for more than 12 months. After discharge, the patients were investigated by telephone and clinic every 2 months, and the complications of patients during this period were counted.

### 2.4. Statistical Analysis

SPSS 20.0 statistical software was used to analyze the data. Measurement data were expressed as mean ± standard deviation ($\bar{x}$ ± *s*), *t*-test was used for comparison between the two groups, count data was expressed as percentage, and the chi-square test was used for comparison between the two groups. *P* < 0.05 means the difference is statistically significant.

## 3. Results

### 3.1. Analysis of the Surgical Conditions of the Two Groups of Patients

The study found that compared with the control group, the operation time, postoperative landing time, and fracture healing time of the observation group were significantly shortened, intraoperative blood loss was significantly reduced, and the difference between the two groups was statistically significant (*P* < 0.05), as shown in Table 1.

### 3.2. Analysis of the Improvement Effect of Hip Joint Function in the Two Groups of Patients

The study found that compared with the control group, the total effective rate of patients in the observation group was significantly higher, and the difference between the two groups was statistically significant (*P* < 0.05), as shown in Table 2.

### 3.3. Changes of Serum MMPs Levels in the Two Groups of Patients before and after Treatment

The study found that there was no statistical difference in the levels of MMP2, MMP6, and TIMP1 between the two groups before treatment (*P* > 0.05). After treatment, the levels of MMP2, MP6, and TIMP 1 in the two groups of patients were lower than those before treatment, and compared with the control group, the decreases in the observation group were more significant (*P* < 0.05), as shown in Table 3.

### 3.4. Changes of Serum RANKL/OPG Levels in the Two Groups of Patients before and after Treatment

The study found that there was no significant difference in RANKL/OPG between the two groups before treatment (*P* > 0.05). After treatment, OPG level in two groups increased, while RANKL level decreased. Compared with the control group, the change trend in the observation group was more significant (*P* < 0.05), as shown in Table 4.

### 3.5. Changes of Serum Interleukin and C-Reactive Protein Levels in the Two Groups of Patients before and after Treatment

The study found that there was no significant difference in the levels of CRP, IL1**β*,* and IL2 between the two groups before treatment (*P* > 0.05), and the above indicators were significantly decreased after treatment (*P* < 0.05), and compared with the control group, the above indicators of the observation group were decreased more significantly (*P* < 0.05), as shown in Table 5.

The article "Therapeutic Effects of the Proximal Femoral Nail for the Treatment of Unstable Intertrochanteric Fractures" was published in 2022. Journal: Evid Based Complement Alternat Med.

### 3.6. Complications

No serious complications occurred in the two groups after treatment.

## 4. Discussion

Elderly unstable femoral intertrochanteric fracture is a common clinical disease and frequently occurring disease, which brings a heavy burden to patients and families. Currently, surgery is usually used for the treatment of femoral intertrochanteric fractures. In this study, it was found that the clinical effect of the proximal femoral antirotation intramedullary nail was better. It is suggested that the proximal antirotation intramedullary nail has a good therapeutic effect on elderly patients with unstable femoral intertrochanteric fracture, and the recovery of MMP and OPG/RANKL levels may be related to the treatment process. Although it is generally believed that proximal femoral anti-rotation intramedullary nails and locking compression plates affect the efficacy of unstable intertrochanteric fractures mainly due to biomechanical rather than biological factors, through this study we confirmed that biological factors, especially changes in the levels of MMPs and their inhibitors, may be involved in the above-mentioned treatment process.

The abnormal expression of MMPs and their inhibitors is involved in the pathological process of a variety of bone tissues and is closely related to the clinical treatment effects [8]. Many clinical medications for bone or joint diseases achieve their therapeutic effects by interfering with MMP levels. Both Polygonatum preparation and celecoxib can improve the joint function score of patients and knee joint function by reducing the content of MMP-13 in their serum, and the reduction of MMP-13 is also related to reducing inflammatory responses and protecting chondrocytes [9, 10]. Drug treatment of knee osteoarthritis can effectively reduce the levels of inflammatory factors such as serum metalloproteinases, thereby improving knee joint mobility and quality of life [11]. When calcitriol is used in the treatment of knee osteoarthritis, it can inhibit MMP by inhibiting MMP-1, MMP-3, and MMP-13 gene expression, thereby reducing the severity of arthritis in patients, reducing pain in patients, and improving the living conditions of patients [12]. This study also found that the levels of MMP2, MMP6, and their inhibitor TIMP1 were significantly reduced in the two groups after treatment, and compared with the control group, the above indicators in the observation group changed more significantly, suggesting that the better therapeutic effect of the proximal bone antirotation intramedullary nail on elderly patients with unstable intertrochanteric fractures may be related to the regulation of abnormal levels of MMPs. Therefore, in addition to the influence of biomechanical factors, biological factors, especially MMPs and their inhibitors, play a key role in the effect of the proximal femoral antirotation intramedullary nail and locking compression plate on the efficacy of unstable intertrochanteric fractures. However, the changes in the above cytokines in patients treated with the proximal femoral antirotation intramedullary nail were more obvious than in those treated with a locking compression plate. Although the changes of the above factors were analyzed in this paper, the regulatory pathways upstream of these factors have not been effectively explored. Future work will focus on the analysis of changes from upstream cytokines.

The article "Therapeutic Effects of the Proximal Femoral Nail for the Treatment of Unstable Intertrochanteric Fractures" was published in 2022. Journal: Evid Based Complement Alternat Med.

The occurrence, development, and treatment of many bone and joint diseases are related to MMPS, RANKL, and OPG. Yougui Pill can delay cartilage degeneration by inhibiting the activity of MMPs and the expression of inflammatory factors. The RANKL/OPG signaling pathway is also closely related to the process of bone metabolism [13, 14]; the effect of traditional Chinese medicine treatment on the levels of serum OPG and RANKL in patients with rheumatoid arthritis of the wind-cold-dampness-type is the key to clinical efficacy [15]. Serum RANKL and OPG levels in patients with ankylosing spondylitis (AS) are significantly correlated with enthesopathy, and they can be used as reliable indicators for predicting the presence of enthesopathy in AS patients, especially the presence of bone erosion [16]. At the same time, percutaneous vertebroplasty can effectively treat senile osteoporotic thoracolumbar fractures and can also significantly reduce the levels of OPG and RANKL and promote bone healing [17]. In this study, after treatment, the levels of RANKL in the two groups were significantly decreased and the level of OPG was significantly increased, indicating that the proximal bone antirotation intramedullary nail has a good therapeutic effect on elderly patients with unstable femoral intertrochanteric fractures, and its effect may be related to the regulation of abnormal levels of MMPs and OPG. Previous studies have also found that interleukin and C-reactive protein are also closely related to the pathology and recovery process of fractures [18, 19]. Incision infection after calcaneal fracture affects the clinical treatment effect, and serum IL-2, IL-6, and CRP levels increase in patients with postoperative incision infection after bone fracture [20]. Closed negative pressure drainage combined with astragalus injection irrigation in the treatment of traumatic suppurative osteomyelitis can effectively improve the patient's limb function, improve treatment efficiency, and reduce complications and hospitalization costs, which may be related to the inhibition of CRP and IL-6 secretion [21, 22]. At the same time, the abnormal recovery of interleukin and C-reactive protein levels has a certain correlation with the recovery of fractures [23–26]. Lugua polypeptide can increase bone mineral density, improve red blood cell-related, bone metabolism and inflammatory indexes in patients with osteoporotic fractures [27], the increase of serum IL-6 level is involved in the injury of elderly femoral neck fracture and acute trauma in the early stage of surgery, and inflammatory response participates in the bone remodeling of postoperative fracture healing [28]. This study also confirmed that the levels of interleukin and CRP in the two groups of patients were significantly reduced after treatment, and the changes in the above indicators in the observation group were more obvious, suggesting that the proximal bone antirotation intramedullary nail is more effective in regulating the abnormally elevated inflammation level in elderly patients with unstable femoral intertrochanteric fractures, which may be related to the regulation of abnormal levels of MMPs and OPG. In future studies, we will further analyze whether MMPs and OPG are risk factors for unstable intertrochanteric fractures and analyze the correlation between them, so as to provide a reference for clinically relevant disease prevention and treatment.

The article "Therapeutic Effects of the Proximal Femoral Nail for the Treatment of Unstable Intertrochanteric Fractures" was published in 2022. Journal: Evid Based Complement Alternat Med.

In conclusion, the proximal femoral antirotation intramedullary nail has a good therapeutic effect on elderly patients with unstable intertrochanteric fractures, and the changes in MMPs and OPG levels may be related to the treatment process.

## Figures and Tables

**Table 1:** Analysis of the surgical conditions of the two groups of patients.

Group	*n*	Operation time (min)	Intraoperative blood loss (ml)	Postoperative landing time (d)	Fracture healing time (weeks)
Control group	*n* = 50	78.43 ± 10.44	116.56 ± 12.56	10.43 ± 1.43	13.34 ± 3.21
Observation	*n* = 50	49.56 ± 9.56^a^	97.21 ± 8.48^a^	6.68 ± 1.90^a^	11.19 ± 3.09^a^
Groupt		1.865	2.334	1.762	1.856
*P*		<0.05	<0.05	<0.05	<0.05

*Note.* Compared with the control group, ^a^*P*<0.05.

**Table 2:** Analysis of the improvement effect of hip joint function in the two groups of patients.

Group	*n*	Cured	Significantly effect	Valid	Invalid	Total efficiency (%)
Control group	50	17	10	18	5	45 (90.0%)
Observation group	50	22	14	13	1	49 (98.0%)
*X * ^2^						2.996
*P*						<0.05

**Table 3:** Changes of serum MMP levels in the two groups of patients before and after treatment.

Group		MMP2 (mg/L)	MMP6 (mg/L)	TIMP1 (mg/L)
Control group (*n* = 50)	Before treatment	34.52 ± 9.23	24.76 ± 5.60	23.65 ± 7.12
	After treatment	29.45 ± 7.09^b^	19.78 ± 4.81^b^	19.60 ± 4.65^b^

Observation group (*n* = 50)	Before treatment	35.09 ± 10.11	25.01 ± 6.33	23.98 ± 8.33
	After treatment	25.53 ± 4.59^ab^	14.54 ± 4.62^ab^	14.36 ± 3.35^ab^

*Note.* Compared with the control group in the same period, ^a^*P*<0.05; compared with before treatment, ^b^*P* < 0.05.

**Table 4:** Changes of serum RANKL/OPG levels in the two groups of patients before and after treatment.

Group		OPG (ng/L)	RANKL (ng/L)
Control group (*n* = 50)	Before treatment	301.33 ± 32.76	14.47 ± 3.88
	After treatment	335.76 ± 27.89^b^	11.09 ± 4.21^b^

Observation group (*n* = 50)	Before treatment	300.98 ± 19.88	15.01 ± 4.09
	After treatment	387.95 ± 25.66^ab^	8.13 ± 1.44^ab^

*Note.* Compared with the control group in the same period, ^a^*P*<0.05; compared with before treatment, ^b^*P* < 0.05.

**Table 5:** Changes of serum CRP, IL1*β,* and IL2 levels in the two groups of patients before and after treatment.

group		CRP (mg/L)	IL1*β* (ng/L)	IL2 (ng/L)
Control group (*n* = 50)	Before treatment	54.54 ± 7.66	47.87 ± 9.44	51.43 ± 8.89
	After treatment	43.43 ± 6.89^b^	40.54 ± 5.21^b^	43.56 ± 7.33^b^

Test group (*n* = 50)	Before treatment	54.09 ± 7.32	48.01 ± 8.33	52.01 ± 9.21
	After treatment	25.64 ± 4.22^ab^	33.13 ± 5.65^ab^	32.34 ± 6.66^ab^

*Note.* Compared with the control group in the same period, ^a^*P*<0.05; compared with before treatment, ^b^*P* < 0.05.

## Data Availability

The raw data supporting the conclusion of this article will be available by the authors without undue reservation.
